The article "Suppression of pancreatic adenocarcinoma upregulated factor (PAUF) increases the sensitivity of pancreatic cancer to gemcitabine and 5FU, and inhibits the formation of pancreatic cancer stem like cells" was published in 2017. Journal: Oncotarget.

# Suppression of pancreatic adenocarcinoma upregulated factor (PAUF) increases the sensitivity of pancreatic cancer to gemcitabine and 5FU, and inhibits the formation of pancreatic cancer stem like cells

**DOI:** 10.18632/oncotarget.19458

**Published:** 2017-07-22

**Authors:** Jae Hee Cho, Sun A. Kim, Soo Been Park, Hee Man Kim, Si Young Song

**Affiliations:** ^1^ Division of Gastroenterology, Department of Internal Medicine, Yonsei University College of Medicine, Seoul, Republic of Korea; ^2^ Division of Gastroenterology, Department of Internal Medicine, Gachon University Gil Medical Center, Incheon, Republic of Korea; ^3^ Division of Gastroenterology and Hepatology, Department of Internal Medicine, Yonsei University Wonju College of Medicine, Wonju, Republic of Korea; ^4^ Brain Korea 21 Project for Medical Science, Yonsei University College of Medicine, Seoul, Republic of Korea

**Keywords:** cancer stem cells, PAUF, pancreatic cancer, MRP5, RRM2

## Abstract

Pancreatic cancer stem cells (CSCs) play a crucial role in tumorigenesis and chemoresistance of pancreatic ductal adenocarcinoma. Pancreatic adenocarcinoma up-regulated factor (PAUF), a novel secretory protein, has been shown to contribute to cancer progression and metastasis. Because the clinical relationship between PAUF and pancreatic CSCs is largely unknown, we investigated the associations between the functional role of PAUF and pancreatic CSCs. Pancreatic cancer sphere cultured from the CFPAC-1 cells showed elevated expression of PAUF and pluripotent stemness genes (Oct4, Nanog, Stat3, and Sox2), and the mRNA of PAUF were increased in CD44^+^CD24^+^ESA^+^ pancreatic CSCs. PAUF knockdown (shPAUF) CFPAC-1 diminished the number of spheres and decreased stemness genes and CSC surface markers (CD133, c-MET and ALDH1). In addition, siPAUF CFPAC-1 decreased the mRNA expression of multidrug resistant protein 5 (MRP5) and ribonucleotide reductase M2 (RRM2) and were more vulnerable to gemcitabine and 5-FU than negative control (p<0.05). In conclusion, PAUF was increased in pancreatic CSCs and the suppression of PAUF enhances chemotherapeutic response to gemcitabine and 5FU by decreasing MRP5 and RRM2 in pancreatic cancer cells.

## INTRODUCTION

Pancreatic ductal adenocarcinoma (PDAC) is one of the most aggressive malignancies and is the fourth leading cause of cancer-related death in the western world [1, 2]. The difficulty in early detection of PDAC and its resistance to conventional treatment options contribute to its dismal prognosis, as indicated by an overall 5-year survival rate of less than 10% [1, 2]. Many researchers have attempted to elucidate the pathogenesis and carcinogenesis of PDAC. However, the molecular basis for the aggressive nature of PDAC is incompletely understood, and the overall survival of patients has not improved significantly despite advances in treatment modalities and introduction of novel targeted therapies.

The article "Suppression of pancreatic adenocarcinoma upregulated factor (PAUF) increases the sensitivity of pancreatic cancer to gemcitabine and 5FU, and inhibits the formation of pancreatic cancer stem like cells" was published in 2017. Journal: Oncotarget.

The clinical outcomes of PDAC may be poor because conventional therapies are directed at tumor cells that have limited tumorigenic potential instead of targeting the pancreatic cancer stem cells (CSCs) that have been identified in human PDAC [3]. Pancreatic CSCs are identified by a variety of biomarkers, and transplantation assays using immune-deficient mice show that pancreatic CSCs self-renew and propagate the parental tumor. Li et al. has identified populations of CSCs in PDAC that express the cell surface markers CD44^+^CD24^+^ESA^+^or c-Met [3, 4]. Apart from these markers, CD133^+^ and ALDH1 are regarded as other markers of CSCs in PDAC [5–7]. These CSCs are also characterized by their chemoresistance, as CD133^+^ pancreatic cancer cells have greater drug resistance to gemcitabine [6], and c-MET inhibitors have been shown to enhance antitumor effects in combination with gemcitabine [3].

Genome-wide analyses have uncovered pancreatic adenocarcinoma up-regulated factor (PAUF), a novel secretory protein associated with pancreatic cancer [8]. Although the mechanism through which PAUF contributes to cancer progression is not clearly established, previous reports suggest it plays critical roles in PDAC progression and metastasis processes, including cell proliferation and modulation of adhesion, migration, and invasion [9–15].

No studies have investigated the association between PAUF and CSCs and how it may contribute to drug sensitivity and resistance. Therefore, the purpose of the present study was to investigate the relationship between PAUF function and pancreatic CSCs. Our experiments provided evidence of PAUF expression in pancreatic CSCs and suggested that PAUF may contributes to multi-drug resistance in the pancreatic CSCs.

## RESULTS

### Pancreatic cancer spheres cultured from human pancreatic cancer cell lines

We used sphere culture to identify CSCs. This *in vitro* method involved culturing candidate pancreatic CSCs with serum-free media containing only EGF and bFGF under nonadherent conditions, and the resulting spheres indicated self-renewal consistent with a CSC phenotype. In this study, PDAC spheres cultured from the CFPAC-1 cells showed upregulated expression of the pluripotent stemness genes Oct4, Nanog, Stat3, and Sox2 relative to adherent CFPAC-1 cells (Figure 1A).

**Figure 1:** PAUF overexpression in pancreatic cancer spheres **(A)** RT-PCR showed that the overexpression of Oct4, Nanog, Stat3, and Sox2 genes in sphere formed from CFPAC-1 cells compare with adherent cells. **(B)** Up-regulation of secretory PAUF was determined by western blot in CFPAC-1, CAPAN-1 and HPAC spheres (Sp) than adherent (Ad) cells.

The article "Suppression of pancreatic adenocarcinoma upregulated factor (PAUF) increases the sensitivity of pancreatic cancer to gemcitabine and 5FU, and inhibits the formation of pancreatic cancer stem like cells" was published in 2017. Journal: Oncotarget.

### PAUF overexpression in pancreatic CSCs

We previously reported PAUF as a novel secretory protein associated with pancreatic cancer [8]. To show the relationship between the PAUF and pancreatic CSCs, secretory PAUF expression were detected in spheres and adherent CFPAC-1 cells by western blot analysis. As Figure 1B, PAUF expressions were upregulated in spheres than adherent CFPAC-1 cells. Furthermore, in other pancreatic cancer cells such as CAPAN-1 and HPAC cells, PAUF expression were upregulated in spheres than adherent cells (Figure 1B).

One of the other enrichment methods of CSCs is fluorescence-activated cell sorting (FACS) through cell surface marker. Based on previous reports that identified the cell surface markers CD44^+^CD24^+^ESA^+^ in a CSC population of human PDAC, we sorted the CFPAC-1 cell line into CD44^+^CD24^+^ESA^+^ and CD44^-^CD24^-^ESA^-^ cells using FACS (Figure 2A), and validated that the previous reported stemness gene expression level using RT-PCR (Figure 2B). Oct4, Nanog, Stat3, Sox2, CD133, c-Met, beta-catenin et al. genes expression levels were upregulated in CD44^+^CD24^+^ESA^+^ than in CD44^-^CD24^-^ESA^-^ CFPAC-1 cells. As well as, PAUF mRNA content was higher in CD44^+^CD24^+^ESA^+^ than in CD44^-^CD24^-^ESA^-^ CFPAC-1 cells (Figure 2B, 2C). Furthermore, in the other pancreatic cancer cell line of HPAC, the expressions of stemness related genes and PAUF were upregulated in CD44^+^CD24^+^ESA^+^ than in CD44^-^CD24^-^ESA^-^ HPAC cells (Figure 2D, 2E).

**Figure 2:** PAUF overexpression in CD24+/CD44+/ESA+ pancreatic CSCs **(A)** CFPAC-1 cells were sorted using surface marker antibodies. CD24^+^/CD44^+^/ESA^+^ cells were 46% and CD24^-^/CD44^-^/ESA^-^ cells were 52%. **(B)** RT-PCR demonstrated that the mRNA expression of stemness-related genes and PAUF was higher in CD24^+^/CD44^+^/ESA^+^ pancreatic CSCs sorted from CFPAC-1 cells than in CD24^-^/CD44^-^/ESA^-^ CFPAC-1 cells. **(C)** Bar graph demonstrated that quantitative analysis of RT-PCR data. **(D)** HPAC-1 cells were sorted using surface marker antibodies. CD24^+^/CD44^+^/ESA^+^ cells were 19.1% and CD24^-^/CD44^-^/ESA^-^ cells were 19.2%. **(E)** RT-PCR demonstrated that the mRNA expression of stemness-related genes and PAUF was higher in CD24^+^/CD44^+^/ESA^+^ pancreatic CSCs sorted from HPAC-1 cells than in CD24^-^/CD44^-^/ESA^-^ HPAC-1 cells. **(F)** Bar graph demonstrated that quantitative analysis of RT-PCR data.

### PAUF knockdown effects on pancreatic cancer stem cells in pancreatic cancer cell lines

To further access the specific role of PAUF in pancreatic CSCs function, we stably knocked down PAUF expression using shRNA targeting regions of PAUF.(Figure 3A) The shPAUF CFPAC-1 cells showed reduced cell proliferation, migration ability and *in vivo* xenograft tumor formation. Migration ability also decreased 0.67-fold in shPAUF CFPAC-1 cells compared with NC CFPAC-1 cells (mean ± SD); 187.71 ± 41.33 cells/microscopic field in shPAUF vs. 278.67 ± 28.66 cells/microscopic field in NC (Figure 3B). To investigate the effect of PAUF knockdown on the xenograft tumor formation *in vivo*, both shPAUF and NC CFPAC-1 cells were injected subcutaneously into nude mice. After 48 days, shPAUF CFPAC-1 cells formed 0.44-fold smaller tumor compared with NC CFPAC-1 cells (mean ± SD); the average tumor size was 114.5 ± 30.12 mm^3^ in shPAUF-xenografts vs. 258.0 ± 103.0 mm^3^ in NC-xenograft mice (Figure 3C). The effect of PAUF knockdown on CSCs-related characteristics was determined using sphere formation and soft agar assay. The number of sphere formation was markedly diminished in shPAUF CFPAC-1 cells compared with NC CFPAC-1 cells. (Figure 3D). Furthermore, the soft agar assay showed that the number of colonies was also 0.54-fold lower in the shPAUF CFPAC-1 cells (mean ± SD); 106.25 ± 0.24 colonies in shPAUF vs. 195.25 ± 0.10 colonies in NC (Figure 3E).

The article "Suppression of pancreatic adenocarcinoma upregulated factor (PAUF) increases the sensitivity of pancreatic cancer to gemcitabine and 5FU, and inhibits the formation of pancreatic cancer stem like cells" was published in 2017. Journal: Oncotarget.

**Figure 3:** PAUF knockdown effects on pancreatic cancer stem cells in pancreatic cancer cell lines **(A)** PAUF knockdown CFPAC-1 cells were established by shRNA transfection, and shPAUF CFPAC-1 cells were confirmed using RT-PCR and western blot. B-actin and GAPDH served as a loading control. **(B)** Migration assays showed that shPAUF CFPAC-1 cells had decreased migration ability compared with NC CFPAC-1 cells; 187.71 ± 41.33 cells/microscopic field in shPAUF vs. 278.67 ± 28.66 cells/microscopic field in NC **(C)** *in vivo* tumor cell xenograft assay showed shPAUF CFPAC-1 cells formed smaller size of tumor compared with NC CFPAC-1 cells; the average tumor size 114.5 ± 30.12 mm^3^ in shPAUF vs. 258.0 ± 103.0 mm^3^ in NC. **(D)** Sphere formation assays showed that shPAUF CFPAC-1 cells had a lower sphere-forming ability compared with NC CFPAC-1 cells. **(E)** Soft agar assays showed that shPAUF CFPAC-1 cells had lower number of colonies compared with NC CFPAC-1 cells; 106.25 ±0.24 colonies in shPAUF vs. 195.25 ± 0.10 colonies in NC **(F)** RT-PCR demonstrated that the expression of pluripotent stemness genes and cancer stem cell-related genes were reduced in shPAUF CFPAC-1 cells compared with NC CFPAC-1 cells. **(G)** Western blot showed a lower protein expression of PAUF and cancer stem cell-related proteins in shPAUF CFPAC-1 cells compared with NC CFPAC-1 cells.

The article "Suppression of pancreatic adenocarcinoma upregulated factor (PAUF) increases the sensitivity of pancreatic cancer to gemcitabine and 5FU, and inhibits the formation of pancreatic cancer stem like cells" was published in 2017. Journal: Oncotarget.

The mRNA and protein expression of pluripotent stemness genes in shPAUF CFPAC-1 was measured using RT-PCR and western blot, respectively. The expression of stemness-related genes (including Oct4, Nanog, and Sox2), and CSC surface markers (such as CD44, CD133, and c-Met) were lower in the shPAUF CFPAC-1 than in the control CFPAC-1 cells (Figure 3F). Protein expression of PAUF, Sox2, and ALDH were lower in shPAUF CFPAC-1 than in control cells (Figure 3G).

### Effects of PAUF on chemoresponse of pancreatic cancer cell lines

Past studies have suggested that pancreatic CSCs are more resistant to anti-cancer chemotherapy agents such as gemcitabine and 5-FU. To determine the role of PAUF in chemoresponse, we performed cell survival assays to validate cytotoxic effects of 5-FU or gemcitabine against PAUF-associated pancreatic cancer. Two transient siPAUF RNAs were used for this experiment.

Both siPAUF CFPAC-1 and siPAUF cells were more vulnerable to the two cytotoxic drugs than the control CFPAC-1 cells (p<0.05, Figure 4A–4B). Furthermore, mRNA expression of PAUF, multidrug resistant protein 5 (MRP5) and ribonucleotide reductase M2 (RRM2) was lower in siPAUF CFPAC-1 cells than in control cells (Figure 4C). These responses for knockdown effect of PAUF were in same manner in AsPC-1 cells (Figure 4D–4F).

**Figure 4:** Effects of PAUF on chemoresponse of pancreatic cancer cell lines **(A-B)** PAUF knockdown effects on the cytotoxicity of 72 hours inoculation with gemcitabine and 5FU in CFPAC-1 cells. MTT assay showed significantly increased antitumor effect of gemcitabine (A) and 5FU (B) in PAUF-silenced CFPAC-1 cells compared with negative control CFPAC-1. Data are shown as the mean ± SD. **(C)** RT-PCR demonstrated mRNA expression of MRP5 and RRM2 was lower in the siPAUF CFPAC-1 cells than in the negative control CFPAC-1 cells. **(D-E)** PAUF knockdown effects on the cytotoxicity of 72 hours inoculation with gemcitabine and 5FU in AsPC-1 cells. MTT assay showed significantly increased antitumor effect of gemcitabine (D) and 5FU (E) in PAUF-silenced AsPC-1 cells compared with negative control CFPAC-1. **(F)** RT-PCR demonstrated mRNA expression of MRP5 and RRM2 was lower in the siPAUF AsPC-1 cells than in the negative control AsPC-1 cells

## DISCUSSION

Recent studies have demonstrated the presence of pancreatic CSCs, which are capable of self-renewal and production of differentiated progeny, in PDAC. Although the isolation and culturing of pancreatic CSCs remains difficult, the role of CSCs in development, maintenance, and metastasis of PDAC is increasingly recognized. In this study, we cultured the pancreatic cancer cells in serum-free media and obtained pancreatic cancer sphere cells, which had self-renewal capabilities. Relative to the adherent cells, PDAC spheres showed increased mRNA and protein expression of PAUF and the pluripotent stemness genes Oct4, Nanog, Sox2 and STAT3. Additionally, CD44^+^CD24^+^ESA^+^ pancreatic CSCs had increased mRNA expression of PAUF.

The article "Suppression of pancreatic adenocarcinoma upregulated factor (PAUF) increases the sensitivity of pancreatic cancer to gemcitabine and 5FU, and inhibits the formation of pancreatic cancer stem like cells" was published in 2017. Journal: Oncotarget.

We recently identified PAUF, (also known as a paralog of ZG16B), a novel 27-kDa secretory protein highly expressed in human PDAC [8]. As an autocrine factor, PAUF is involved in altered migration, invasion, proliferation, and metastasis [9, 11, 16]. PAUF also acts as a paracrine factor by causing stromal changes in the tumor microenvironment that promotes tumor evasion of the immune surveillance system [12]. PAUF also modulates permeability of the endothelial cells and vasculature to promote tumor angiogenesis [17]. Although only a few preclinical studies have investigated anti-PAUF monoclonal antibodies, PAUF-specific RNA aptamers (P12FR2), and adenoviral PAUF-targeting trans-splicing ribozymes (TSR) for PDAC, PAUF-targeted therapies may be an alternative approach for cancer treatment [10, 14, 15]. The above-mentioned studies suggest functional roles of PAUF in pancreatic cancer; however, little is known about the clinical relationship between PAUF and pancreatic CSCs. Therefore, we show the association between PAUF expression and characteristics of CSCs to determine the contribution of PAUF activity to chemoresponse in pancreatic CSCs,

Of clinical importance, recent research suggests CSCs are resistant to conventional chemotherapy and radiation [4]. Enhanced expression of ATP-binding cassette (ABC) family of transporters has been shown to be characteristic of side population cells with CSC features. These side population cells are more resistant to chemotherapeutic agents and may play a key role in tumor progression, recurrence, and metastasis [18, 19]. To identify the relationship between chemoresponse and the functional role of PAUF, we conducted cytotoxic studies with gemcitabine and 5-FU in siPAUF CFPAC-1/siPAUF AsPC-1 cells and negative controls. Our study showed that siPAUF CFPAC-1/siPAUF AsPC-1 cells were significantly more vulnerable to both cytotoxic drugs. Similar to our results, recent study reported that silencing of PAUF leads to increase the sensitivity to gemcitabine in BxPC-3 cells and this mechanism may involve drug transporter such as MRP2, MRP3, and MDR1 genes [20]. However, because both chemosensitivity and chemoresistance can occur through intracellular enzymes regardless of drug transporters, we measured the mRNA expression of genes involved in drug metabolism (such as dCK, CDA, RRM1, and RRM2) in addition to transporters (including MRP3, MRP4, MRP5, and hENT1). In the present study, the both siPAUF CFPAC-1 and siPAUF AsPC-1 cells decreased mRNA expression of MRP5 and RRM2. MRP5 (also known as ABCC5) is a member of the multidrug resistance-associated protein subfamily of ABC transporters and confers resistance against chemotherapeutic drugs such as etoposide, 5-FU, and gemcitabine [21–23]. RRM2 is the catalytic subunit of ribonucleotide reductase, a dimeric enzyme that supplies deoxynucleotides essential for DNA replication and cell growth. The overexpression of RRM2 has been associated with gemcitabine resistance and increased cellular invasiveness *in vitro* [24], [25] and high expression of RRM2 in pancreatic tumors is associated with reduced overall survival after resection [26].

The article "Suppression of pancreatic adenocarcinoma upregulated factor (PAUF) increases the sensitivity of pancreatic cancer to gemcitabine and 5FU, and inhibits the formation of pancreatic cancer stem like cells" was published in 2017. Journal: Oncotarget.

Taken together, our study indicated that PAUF signaling was required for the formation of pancreatic CSCs. In addition, the suppression of PAUF may contribute to increase drug sensitivity through mechanisms involving MRP5 and RRM2, thus making it a novel target for treatment of PDAC. However, our study had some limitations. First, we could not demonstrate a PAUF mediated signal transduction mechanism by which PAUF induces CSCs phenotypes. Second, we used pancreatic cancer cell lines rather than patient-derived pancreatic cancer cells and only investigated the effect of PAUF knockdown in PDAC cancer cell lines rather than in pancreatic CSCs derived from human tissues. Third, we did not perform the experimental study using *in vivo* models of human PDAC, which are required to prove a causal relationship between PAUF and target proteins such as MRP5 and RRM2. Thus, the possible connection between PAUF, drug transporters, and cell signaling pathways should be investigated in future studies.

In conclusion, we showed that PAUF is a novel protein overexpressed in human pancreatic CSCs that may contribute to chemosensitivity by decreasing MRP5 and RRM2. Thus, PAUF may constitute a therapeutic target to enhance the drug sensitivity of pancreatic CSCs.

## MATERIALS AND METHODS

### Cell culture

Four PDAC cell lines (AsPC-1, Capan-1, CFPAC-1, and HPAC) were obtained from ATCC(American Type Culture Collection). All cells were grown in the appropriate conditioned medium and maintained in an atmosphere of 5% CO_2_/95% air at 37°C. We primarily used CFPAC-1, which expresses high endogenous levels of PAUF, for our experiments. In order to form cancer spheres, single cells were cultured for 7 days in Dulbecco's Modified Eagle Medium: Nutrient Mixture 12 (DMEM/F12,1:1; Gibco) containing 0.5% fetal bovine serum (FBS) (Hyclone), 0.5% bovine serum albumin fraction V (Gibco), insulin-transferrin-selenium A (Gibco), 10 ng/ml human epidermal growth factor (hEGF; R&D systems, Wiesbaden-Nordenstadt, Germany), 10 ng/ml human fibroblast growth factor (hFGF; R&D), and 10 ng/ml human leukemia inhibitory factor (hLIF; R&D) at a density of 1×10^3^ cells/ml in an ultralow attachment plate (Corning, Corning, NY, USA). Growth factors were added every 3 days. For preparation of secretory proteins, culture medium was changed to serum-free medium in the post sphere culture after 5 days and cultured for an additional 2 days.

The article "Suppression of pancreatic adenocarcinoma upregulated factor (PAUF) increases the sensitivity of pancreatic cancer to gemcitabine and 5FU, and inhibits the formation of pancreatic cancer stem like cells" was published in 2017. Journal: Oncotarget.

### Semi-quantitative PCR (reverse transcription PCR)

The total RNA from cancer cells was extracted using a RNA easy extraction kit (Qiagen) according to the manufacturer's instructions. To quantify the relative expression of the genes, we used β-actin primer as a control. The PCR primers used were PAUF sense, 5’-cacctgggcagggaagatgta-3’; PAUF antisense, 5’-gctcagtggtcggctcctct-3’; β-actin sense, 5’-ggcatc ctcaccctgaagta –3’; and β-actin antisense, 5’-ggggtgttgaa ggtctcaaa-3’. The PCR primer sequences for the expression of genes related to pancreatic CSCs are described in Table 1.

**Table 1:** The sequences of PCR primer for the expression of known pancreatic CSCs related molecules

Name	Sequence
ß-catenin (sense)	GTATGAGTGGGAACAGGGATTT
ß-catenin (antisense)	CCTGGTCCTCGTCATTTAGC
SOX2 (sense)	CACAACTCGGAGATCAGCAA
SOX2 (antisense)	GTTCATGTGCGCGTAACTGT
NANOG (sense)	ACTGTCTCTCCTCTTCCTTCCT
NANOG (antisense)	AGAGTAAAGGCTGGGGTAGGTA
OCT4 (sense)	AAG TGG GTG GAG GAA GCT
OCT4 (antisense)	CGA GGA GTA CAG TGC AGT
STAT3 (sense)	GTCTGGCTGGACAATATCAT
STAT3 (antisense)	TTGGGAATGTCAGGATAGAG
CD44 (sense)	CACCATTTCAACCACACCAC
CD44 (antisense)	GGTGTTGTCCTTCCTTGCAT
CD133 (sense)	GCTCAGACTGGTAAATCCCC
CD133 (antisense)	GACTCGTTGCTGGTGAATTG
c-MET (sense)	CAA TGT GAG ATG TCT CCA GC
c-MET (antisense)	CCT TGT AGA TTG CAG GCA GA
ALDH1A1 (sense)	AGCAGGAGTGTTTACCAAAGA
ALDH1A1 (antisense)	CCCAGTTCTCTTCCATTTCCAG
ABCG2 (sense)	CAC TGA TCC TTC CAT CTT GT
ABCG2 (antisense)	TAT GAG TGG CTT ATC CTG CT

### Establishment of stable PAUF knockdown cell line using shRNA

The shRNA-expressing plasmid targeting human PAUF and negative control plasmid were purchased from SABiosciences. The human PAUF shRNA sequence was 5’-ACACCAGCAAGGACCGCTATT -3’ and the control shRNA sequence 5’-GGAATCTCATTCGATGCATAC -3’. For shRNA transfection, CFPAC-1 cells were plated into 6-well plates at a density of 5×10^4^ cells/well the day before transfection. Transfection was performed using Lipofectamine2000 reagent according to manufacturer's instructions, and stable knockdown clones were selected using neomycin.

The article "Suppression of pancreatic adenocarcinoma upregulated factor (PAUF) increases the sensitivity of pancreatic cancer to gemcitabine and 5FU, and inhibits the formation of pancreatic cancer stem like cells" was published in 2017. Journal: Oncotarget.

### Transient transfection of small interfering RNA (siRNA) targeted for PAUF

The two sets of 25-nucleotide stealth RNAi-targeting PAUF were synthesized customarily by Invitrogen. Stealth RNAi duplexes, which have a similar GC content to that of the duplex siRNA obtained from Invitrogen, were used as negative controls. Stealth RNAi-targeting PAUF were transfected into CFPAC-1 cells using Lipectamine™ RNAi Max transfection agent (Invitrogen) according to the manufacturer's protocol. Cells were harvested 72 h post-transfection and subjected to total RNA extraction and a migration and invasion assay. Secreted protein was prepared from culture medium 48 h post-transfection.

### MTT assay

After incubation at 37°C overnight, cells were treated with various concentrations of gemcitabine or fluorouracil (5-FU) in complete growth media and incubated for 72 h at 37°C. A 3-(4,5-dimenthelthiazol-2-ly)-2,5-diphenyltetrasolium bromide-based assay (absorbance 570 nm) was used to measure the number of metabolically active cells.

### Flow cytometry and cell sorting

Cultured cells were detached with accutase solution (Sigma-Aldrich, Inc., St. Louis, MO, USA) and washed in phosphate-buffered saline (PBS) containing 0.5% FBS. Single cells were stained for 20 min on ice in the dark, washed twice in PBS containing 0.5% FBS, and fixed in 2% paraformaldehyde. Flow cytometry analysis was performed using a FACSCalibur system (BS Biosciences, San Jose, CA), and cell sorting was performed using FACSAria II (BD Immunocytochemistry System, Franklin Lakes, NJ). Antibodies against CD24 (anti-CD24-PE, BD), CD44 (anti-CD44-APC, BD), and ESA (anti-ESA-FITC, BD) were used. FITC-mouse IgG2b, κ isotype control (BD), rat IgG1 κ isotype control FITC (eBioscience), PE-mouse IgG2a, κ isotype control (BD), and APC-mouse IgG2b, κ isotype control (BD) were used as controls.

### Protein extraction and western blot

Cells were prepared in lysis buffer containing 50 mM HEPES (pH 7.2), 150 mM NaCl, 25 mM beta-glycerophosphate, 25 mM NaF, 5 mM EGTA, 1 mM EDTA, 1% NP-40, 1 mM sodium orthovanadate, 0.1 mM phenylmethanesulfonylfluoride (PMSF), and a protease inhibitor cocktail (Roche Diagnostics). For secretory protein preparation, culture medium was centrifuged and the cellular components and debris were discarded. Culture medium was concentrated by the addition of ice-cold acetone, and the precipitated protein was resuspended with lysis buffer. Proteins were separated on SDS-PAGE and transferred to 0.45-μm Immobilon P-transfer membrane (Millipore). Membrane was blocked in 5% (w/v) non-fat milk and probed with the following primary antibodies: anti-human PAUF antibody (2009 Cancer Science), Sox2 (Cell Signaling Technology), Oct4 (Cell Signaling Technology), Nanog (Cell Signaling Technology), aldehyde dehydrogenase (ALDH) (BD), Cdk6 (Santa Cruz), cyclin D3 (Santa Cruz), Snail (Cell Signaling Technology), slug (Cell Signaling Technology), twist (Cell Signaling Technology) and glyceraldehyde phosphate dehydrogenase (GAPDH) (Santa Cruz). Immunoreactive material was then visualized using SuperSignal West Pico Chemiluminescence Substrate [27] according to the manufacturer's instructions.

The article "Suppression of pancreatic adenocarcinoma upregulated factor (PAUF) increases the sensitivity of pancreatic cancer to gemcitabine and 5FU, and inhibits the formation of pancreatic cancer stem like cells" was published in 2017. Journal: Oncotarget.

### Soft agar assay

A suspension of 500 single cells containing 0.3% agar medium was overlaid on 0.6% agar medium in 24-well plates. Each well was covered with complete medium, and the plates were incubated for 4 weeks. Colonies were stained with crystal violet and counted. Experiments were done in triplicate.

### Cell proliferation, migration and invasion assay

For cell proliferation, 2 × 10^3^ cells were seeded per sell into 24 well plates. Every 24 h, the number of cells was counted. The experimental was done in triplicate to determine the number of cells at each time point. The migration assays were performed in 6-well Transwell plates (Costar, Cambridge, MA). Cells (1 × 10^5^) were seeded in triplicate in the upper compartment. The media incubated the NIH/3T3 with DMEM for 24 hours was added to the lower wells. Following 24-hour incubation at 37C in a 5% CO_2_ humidified incubator the cells in the upper chamber and on the surface of the filter were completely removed by wiping with a moist cotton swab. Cells that had migrated through the filter and adhered to the outer surface were fixed with methanol and stained with Toluidine Blue. Invading cells were examined, counted and photographed by microscopy at 100× magnification. The invasive abilities were tested by Matrigel invasion assay. Assays were performed in 6-well Transwell plates (Costar, Cambridge, MA) with an 8 μm pore size were coated with Matrigel (Becton Dickinson). Cells (1 × 10^5^) were then seeded in triplicate in the upper compartment chamber coated with Matrigel. The media incubated the NIH/3T3 with DMEM for 24 hours was added to the lower wells. Following 48-hour incubation at 37C in a 5% CO_2_ humidified incubator the cells in the upper chamber and on the surface of the filter were completely removed by wiping with a moist cotton swab. Cells that had invaded the Matrigel, migrated through the filter and adhered to the outer surface were fixed with methanol and stained with Toluidine Blue. Invading cells were examined, counted and photographed by microscopy at 100× magnification.

### *In vivo* tumorigenic assay

Cells were resuspended at a cell density of 3x 10^6^ cells in 150 μl of serum-free culture medium and injected subcutaneously into the BALB/c nude female mice (6 weeks of age). Tumor formation was monitored twice a week measuring the width and length. Tumor volumes were calculated by the formula V (mm^3^) = A x B^2^, where A is the largest dimension and B is the perpendicular diameter. Tumor xenografts were recovered from mice, fixed in 4% paraformaldehyde, and embedded in paraffin.

The article "Suppression of pancreatic adenocarcinoma upregulated factor (PAUF) increases the sensitivity of pancreatic cancer to gemcitabine and 5FU, and inhibits the formation of pancreatic cancer stem like cells" was published in 2017. Journal: Oncotarget.

### Statistical analysis

Mann-Whitney U test and independent *t*-test were used to compare cell survival between siPAUF and control groups. Statistical calculations were performed using SPSS (version 12.0 for Windows; SPSS, Inc., Chicago, IL, USA). Values of *p* < 0.05 were considered statistically significant. For quantitative analysis western blot and RT-PCR data, we used ImageJ softwere (U.S. National Institutes of Health, Bethesda, MD, https://imagej.nih.gov/ij).

## Acronyms list

PDAC: Pancreatic ductal adenocarcinoma
CSCs: Cancer stem cells
PAUF: Pancreatic adenocarcinoma up-regulated factor
Oct4: Octamer-binding transcription factor 4
Stat3: Signal transducer and activator of transcription 3
Sox2: Sex determining region Y-box 2
ESA: Epithelial-specific antigen
ALDH: Aldehyde dehydrogenase
PTEN: Phosphatase and tensin homolog
Lef1: Lymphoid enhancer-binding factor 1
Dvl2: Dishevelled segment polarity protein 2
MRP: Multidrug resistant protein
RRM: Ribonucleotide reductase M
ATCC: American Type Culture Collection
hEGF: Human epidermal growth factor
hFGF: Human fibroblast growth factor
hLIF: Human leukemia inhibitory factor
FACS: Fluorescence-activated cell sorting
CDK6: Cyclin-dependent kinase 6
dCK: Deoxycytidine kinase
ENT1: Equilibrative nucleoside transporter 1
